The article "Practice and Exploration of Music Solfeggio Teaching Based on Data Mining Technology" was retracted in 2023. Reasons: unreliable results or conclusions; concerns about the data; concerns about the peer review; concerns about the citations.

# Practice and Exploration of Music Solfeggio Teaching Based on Data Mining Technology

**DOI:** 10.1155/2022/5436772

**Published:** 2022-08-16

**Authors:** Wenfeng Zhang

**Affiliations:** Liaocheng University Dongchang College, Liaocheng 252000, China

## Abstract

People can learn, understand, and use music using the solfeggio method. People involved in professional music training have given it importance because it is a fundamental discipline of enlightenment music and a necessary training method and technical theory course to enter the professional level. This article presents an in-depth analysis of the music curriculum model based on data mining technology. Additionally, a music style classification method based on FP Growth association rules mining is developed, which decreases the number of frequent element sets needed and speeds up database scanning. To better match the characteristics of music, a multirepetition structure model is used, and the MFCC (Mel-frequency cepstral coefficients) function is used to set the repetition structure model. The results demonstrate that the music style classification method put forth in this article has clear advantages in terms of efficiency: when the minimum support is 0.2 percent, this method's execution time is about 33 percent compared to the other methods. The outcomes of the experiment suggest that this method can more accurately capture the repeatability of music and enhance separation performance to some extent.

## 1. Introduction

Solfeggio is a broad field of study. It involves all facets of music, and its significance in developing the full range of musical talent should not be understated. On the other hand, the teaching goals of some instructors lag behind; the majority only call for students to understand tone and rhythm, oblivious to the students' inner perceptions of their own needs for the practice and only beginning at the surface. Training not only falls short of the intended outcome but also produces dull classroom material [1]. As a result, the roll-call theme is by no means a tool. Closing the music foundation outside of the application programme, creating an independent system, and adhering to a particular, predetermined, and predefined teaching are all impossible.

The main goal of the solfeggio course, which is also a crucial foundation for learning the fundamentals of music, is to gradually develop students' musical senses, including intonation, speed, rhythm, and melody, through the practice of solfeggio. The rating of solfeggio does not appear to be very high. To enhance the learning environment in the classroom, Salaman suggested paying close attention to the use of “original music” along with dance, movements, speech, and other comprehensive teaching methods [2]. In this essay, the author illustrates the training techniques and importance of Orff's music teaching methodology through rhythm, movement, and motivation. Steers serve as the foundation for the solfeggio teaching activities in the classroom. Students' interest in taking this course can be piqued by incorporating the excellent teaching strategy of “Body Rhythm” into senior high school solfeggio lessons [3]. Gilbert discussed a number of solfeggio training tenets in Kodály's teaching approach, which, while useful as a teaching benchmark, lacks any real-world application [4]. Using an experimental report, Kallio and Westerlund [5] presented the practical significance of Kodály's teaching method in terms of enhancing the overall musical quality of primary school students after discussing the viability of localising it. Because everyone has a different level of intelligence, different teaching strategies are needed to foster that diversity. Not only has the theory of multiple intelligences developed into a fundamental tenet of American educational reform, but it also fits the requirements of contemporary Chinese educational development and reform and offers a theoretical framework for implementing high standards of education there.

With the growing use of data mining (DM) technology in the education sector, educators are now required to categorise various research objects, create research models for each type, gather a variety of user data, and then use a variety of algorithms, relational graph models, or music course resource classifiers to create a music expert system based on big data [6, 7]. The expressive singing technique used in solfeggio can help students better understand music and increase their desire to express it. Students' exposure to the arts can help them become familiar with the most well-known songs in the world and improve their musical and artistic abilities. Public education and professional development are integrally linked. The social value of this essay also lies in its investigation of the fusion of humanistic principles and fundamental music education, or, more specifically, in its focus on the fusion of aesthetics and educational objectives.

### 1.1. Innovation

1. The improvement and augmentation of solfeggio instruction are made possible by the effective use of multimedia technology. The uniqueness of conventional teaching methods can be resolved, classroom instruction can be improved, classroom content can be enriched, and teaching methodology can be improved with the proper and thorough application of multimedia technology. In order to improve information services for schools, teachers, and students, this article makes effective use of information media such as databases and educational clouds to thoroughly explore the music curriculum mode based on DM technology.
2. Signal processing includes the processing of music. The study of computer music processing is becoming more and more crucial in order to allow computers and people to freely communicate with music. The music recognition in this article simulates human cognition and computer music analysis by combining the knowledge and technology of computer multimedia technology, signal processing, and pattern recognition with music theory.

## 2. Related Work

### 2.1. Musical Solfeggio

Foreign music education has always been in a leading position. Around the 20th century, foreign music education developed continuously, forming an advanced education system. Chesky believed that teachers should know fairly well the examination form, content, and outline of the art joint entrance examination, and then choose appropriate teaching contents and methods according to the requirements of the examination, and carry out solfeggio teaching targeted at high school music majors, so as to achieve twice the result with half the effort [8]. Hamilton discussed that the purpose of music reading and writing is to cultivate students' all-around ability, deeply analyzed the idea of Kodály's teaching method, and put forward some guiding suggestions for staff teaching in school music teaching [9]. Ma put forward the practical problems of the Kodály teaching method in the solfeggio course [10]. According to the nature of its solfeggio course, it is named “Basic Music Quality,” and this major is named “Basic Music Quality Education Major,” with musical hearing ability as the core of music quality. It can be seen that solfeggio education and teaching are of great value to the cultivation of comprehensive quality.

Tamuro and Kawasoi thought that the discrimination basis, training process, development, application, and evaluation of various intelligences in music solfeggio theory are of great help to the training of various skills in solfeggio and the study of related disciplines [11]. Hausman et al. showed a students' relaxed, harmonious, dynamic space for music learning, which is full of aesthetic feeling and strong human touch so that students will step into the wonderful hall of music art under the guidance of teachers [12]. Colish has added a new subject learning content with a new educational concept, which aims to help students comprehensively apply their existing knowledge and experience, solve challenging and comprehensive problems through independent exploration and cooperation and exchange, and cultivate their problem-solving ability [13]. Mangini's teacher-centered teaching mode, which simply teaches book knowledge, helps students develop the ability to explore knowledge, obtain information and learn independently, encourages students to actively try learning methods such as observation, thinking, induction, and summary, and strengthens the guidance of learning methods so that students can form effective learning strategies.

### 2.2. DM Related Research

From a large number of incomplete, noisy, chaotic, and random practical application data, DM is the process of extracting hidden, unknown, but potentially useful information and knowledge. Based primarily on artificial intelligence, machine learning [14, 15], statistics, and other technologies, the company's original data is analyzed, inferred, and reasoned, potential patterns are extracted, and customer behaviour is predicted, assisting enterprise decision makers to adjust market strategies, reduce risks, and make the right decisions.

Zhang proposed a second-order Markov chain algorithm based on characteristic melody mining, which introduced characteristic melody mining on the basis of association rule mining Apriori algorithm to realize music composition style training [16]. Panwar et al. proposed that the FP_Growth association rule mining algorithm should be applied to the genre classification task of music media, which can effectively improve the database scanning speed without a candidate item set [17]. Wilson et al. proposed some improved kNN (k Nea-rest Neighbor) algorithms to deal with multilabel data methods. These methods firstly find out the *k* nearest neighbors of the sample to be predicted, but they are in the aggregation of the sample label set. A different approach was used [18]. Zhang proposed an algorithm that combines lazy learning and association rule learning methods, and its derivation process will only be generated immediately when forecasting [19]. Laukka et al. combined some existing multilabel classification methods with different modes, such as averaging, threshold selection, and weighted averaging, and achieved better results than a single classifier [20].

Niitsuma et al. successfully designed a fuzzy system for automatically analyzing chords. However, because there are too many individualized elements in music, it is difficult to fully explain them with the existing music theories, so the analysis of chords is only limited to the category of music works of a certain style or a certain era [21]. For underdetermined mixed signals, Yin used the method of estimating the energy spectral density to separate the signal sources and used the beamforming method to separate up to M (M-1) + 1 sound sources sensed by M sensors [22]. Gao et al. thought that multichannel audio can be regarded as the convolution mixed source under the underdetermined condition and put forward a separation algorithm of the probability window model [23]. Das et al. introduced sparse representation into the nonnegative matrix, established a complete sparse dictionary set, and adopted the Newton iteration method, which greatly improved the operation speed [24].

## 3. Methodology

### 3.1. Analysis of the Teaching Mode of Music Solfeggio Based on DM Technology

A fundamental component of music education is solfeggio. Basic information and abilities are covered, including solfeggio, ear training, and fundamental music theory. It is distinguished by a multidisciplinary knowledge structure, mutual penetration, and the fusion of theory and technology. To develop a keen and accurate understanding of musical works, it is important to understand the relationship between the major musical parts and the structure of polyphonic music. The goals of solfeggio practice also include the ability to sing while reading music, as well as the ability to listen for harmony. Additionally, various musical genres, music types, and musical structures also contribute to the colourful and distinctive forms that various musical works present (including period, regional, personal, and other styles of music).

Since music is abstract, the ideas it conveys frequently transcend the limitations of language to become even more profound, potent, and moving. Solfeggio has two main styles: listening and dictation, both of which include single tones, intervals, chords, melodies, and rhythm. If you are listening to a melody, you should be able to determine the melody's regularity and other factors. These sounds and musical compositions are used as symbols in musical performances to convey the qualities of different musical elements that come together to create a complete piece of music. From a psychological perspective, practising the ability to reflect a symbol is very beneficial to mastering the symbol's corresponding ability. The impact of instruction is most strongly influenced by curriculum implementation. Teachers should improve their comprehension of the course concept, content organisation, and training objectives of the solfeggio course. The designers of university curricula must prepare front-line instructors, increase communication, and learn from first-hand experience. The understanding of skills in solfeggio training is biassed. In addition to strengthening classroom supervision and management, we should ask teachers to prepare lessons carefully, put an end to some of their lazy habits, and support them as they implement the solfeggio teaching reform. Finally, we should mentor and assist teachers as they address challenges in their classrooms. Teachers' teaching impact and students' learning impact should be assessed when they run into issues in order to assist them in further improving their teaching level.

Resources for music curricula are not only plentiful but also come from a variety of sources. In order to effectively meet both the actual teaching design and the actual needs of the students, a resource bank must be created for careful consideration when developing the education cloud in its infancy. Create an updated, intelligent, and more effective platform for educational resources to address issues with user data collection, integration, and analysis, uneven distribution, slow update, and decreased sharing [8]. The general architecture of this design is shown in Figure 1.

It has many advantages that not only make it simpler to exchange excellent teaching resources but also better support the development of both teachers and students. Teachers can make adjustments to meet the needs of their students and get the necessary teaching materials they require in real time. The user information database collects information and data from user actions on the user interface, classifies all types of information effectively, and transmits that information to the user model and recommendation system, among other systems, in order to transmit user information and teach the music that users are interested in. This system allowed the user to finally comprehend the goal of real-time interactive music teaching materials. The sound is concentrated at the source of shock because at low-frequency resolution, most of the energy of singing is concentrated on a few individual frequencies, while at high-frequency resolution, the influence of pseudoharmonics on the human voice cannot be ignored. Different from the energy of each overtone, the energy of pseudoharmonics is distributed in the whole frequency range.

The energy distribution of singing voice is assumed to be sparse, so under the above-mentioned restrictive conditions, the segments with consistent similarity are integrated together with *S*_Mel_, and the corresponding segments on the energy spectrum *V* are median filtered to obtain the repeated structure model *S* at the corresponding frame, as shown in the following equation:

(1) $$\begin{array}{c} S\left(i,j\right)=\underset{l\in \left[1,k\right]}{\text{median}}\left\{V\left(i,J_{j}\left(l\right)\right)\right\}, \end{array}$$

where *J*_*j*_=[*J*_1_, *J*_*k*_] represents the group of segments with the same repeatability, *k* represents the number of segments, *i* represents the frequency point, and *j* represents the number of frames.

The extracted features are subjected to similarity operation, and the formula is shown in the following equation:

(2) $$\begin{array}{c} S_{\text{Mel}}\left(j_{a},j_{b}\right)=\frac{\sum_{i=1}^{n}V\left(i,j_{b}\right)}{\sqrt{\sum_{i=1}^{n}V{\left(i,j_{a}\right)}^{2}}\sqrt{\sum_{i=1}^{n}V\left(i,j_{b}\right)}}, \end{array}$$

where *S*_*Mel*_ represents MFCC (Mel-frequency cepstral coefficients) similarity matrix, *i* represents dimension and *n*=40, and *j* represents frame number.

It is the key factor of the main melody music style division, which directly affects the performance of the subsequent classification algorithm and is an important preprocessing link. At present, the typical main melody extraction algorithm is the Skyline melody extraction algorithm. Specifically, the average pitch value $\bar{p_{i}}$ of track *c*_*i*_ is calculated by the following formula:

(3) $$\begin{array}{c} \bar{p_{i}}=\frac{\sum_{j=1}^{n}p_{ij}}{n}, \end{array}$$

where *p*_*ij*_ represents the pitch value of note *j* in track *c*_*i*_; *n* is the number of notes in track *c*_*i*_.

Logistic regression is very suitable for some nonlinear classification problems, but it is only suitable for binary classification problems and gives the classification results and the probability of the results. Because logistic regression is aimed at the binary classification problem, the class label *y*_*i*_ ∈ {0,1}. Its hypothetical function is as follows:

(4) $$\begin{array}{c} h_{\theta }\left(x\right)=\frac{1}{1+\exp\left(-\theta^{T}x\right)}, \end{array}$$

where *θ* represents the parameters of the training model.

The focus of music analysis ability is to master music theory knowledge, such as music theory, harmony, music theory analysis, and music history. The ability of music analysis is to combine these rational and conceptual thoughts with perceptual and abstract thoughts. The training focuses on accurately capturing semitone changes, correctly assigning punctuation and connecting sentences, and expressing intensity from weak to strong according to the fluctuation of melody lines. In the process of solfeggio, targeted training should be given to pitch, rhythm, rest, diacritical marks, accents, dynamic changes, and other factors.

### 3.2. Integration of DM Technology and Solfeggio Teaching

The rhythm of music is closely related to it. Along with teaching students the fundamentals of music, teachers should focus on developing their students' sense of rhythm as they learn the solfeggio. The most common method of instruction for rhythm memory and dictation is to remember the head and tail of the notes in the music score by comparing with the staff. The interference of different notes is thought to be eliminated by helping students learn to memorise music notation through rhythm. So, in order to carry out related teaching activities and effectively increase students' learning efficiency in the pitch training process, teachers can effectively use the gesture teaching method in the Kodály music teaching method.

A crucial component of teaching solfeggio is the use of different voices, which can help students perform and express harmony style, rhythm, sound effects, timbre, and other concepts. The use of DM technology in the practice of multipart music has gradually improved the capacity for music collection and adaptation, as well as the imagination and expressive force in multi-part music. To adapt to different needs in the classroom, educators can use a variety of editing techniques, synthesise resources, and choose from a variety of music clips for online processing. Short sentences and quick songs with rich content are created by combining the sounds of different percussion instruments. Targeted, step-by-step training is implemented to enhance students' musical memory and deepen instruction in accordance with the teaching process and students' practical level.

Apriori association rules mining algorithm needs to constantly build candidate sets and filter candidate sets to extract frequent itemsets, and it also needs to scan the original data many times. When the original data is large, the disk I/O amount is excessive, and the efficiency is relatively low. Therefore, the FP_Growth association rule mining algorithm is applied to the music media style classification task. In the association analysis, the specific expressions of support and trust are as follows:

(5) $$\begin{array}{c} s\left(X⟶Y\right)=\frac{\sigma \left(X\cup Y\right)}{N},\\ c\left(X⟶Y\right)=\frac{\sigma \left(X\cup Y\right)}{\sigma \left(X\right)}, \end{array}$$

where *N* represents the number of transactions.

In this article, the support calculation method of music classification is as follows:

(6) $$\begin{array}{c} s=\left|\left\{x|x\in D,{\text{rule}}_{i}\in x\right\}\right|, \end{array}$$

where *D* represents the training dataset; *rule*_*i*_ is the rule of *D*. Sets are treated as itemsets in association analysis.

The classical HMM (Hidden Markov model) is a model based on statistical signals, which is the most successful and widely used model at present. Although the state of HMM is hidden, in many practical applications, the state of the model often has certain physical significance. Generally speaking, states are interrelated, and any state can be transferred from other states. Part of this should be to analyze the chords of music and extract its features so it does not need a high sampling rate. The specific steps are as follows:

Frame processing divides it into overlapping frames with 4095 sampling points in each frame, followed by STFT (short-time Fourier transform):

(7) $$\begin{array}{c} X_{\text{STFT}}\left(k,n\right)=\sum_{m=0}^{N-1}x\left(n-m\right)\cdot w\left(m\right)\cdot e^{-j2\pi km/N}, \end{array}$$

where *k* represents the frequency coordinate, 0 ≤ *k* ≤ *N* − 1, *n* represents the center of the short-time Fourier transform window, and *w*(*m*) represents the Hanning window of *N*=4095 points.

The mapping from frequency to sound level is calculated logarithmically according to the average law in music theory. Choose a step length of 100 ms, that is, 10 tone profile frames per second. *k* in STFT is mapped to *p* in tone profile. The mapping formula is as follows:

(8) $$\begin{array}{c} p\left(k\right)=\left[10\cdot \;\log_{2}\left(\frac{k}{N}\cdot \frac{f_{sr}}{f_{ref}}\right)\right]\mathrm{mod}10, \end{array}$$

where *f*_*ref*_ is the reference frequency corresponding to tone profile and *f*_*sr*_ is the sampling rate.

A HMM model is a stochastic finite state machine in which each state produces an observation. The transition of its state obeys Markov property, that is, under the condition that its current state is known, its future evolution has nothing to do with the past state—the present and the future are independent of the past. The frame diagram of the string identification system is shown in Figure 2.

Before model training, we first define the topology of HMM and use the ergodic model to determine the transition probability because the transition between any chord states is possible. If you know the observation vector produced by each state for training data, you can directly estimate the model parameters. During the execution of the algorithm, the best state is saved in every step of the recursion process. When the recursion is over, an optimal state transition sequence can be retrieved, thus maximizing the probability of observing the vector and obtaining the best recognition result. As a result, each frame is assigned a string type.

The natural frequency of the system is

(9) $$\begin{array}{c} p_{n}=\frac{n\pi }{l}\sqrt{\frac{T_{0}}{\rho A}},\;n=1,2,\ldots , \end{array}$$

where *T*_0_ represents the tension of the string, *A* represents the cross-sectional area of the string, *ρ* represents the density of the string, *l* represents the length of the string, which is divided into *n*+1 segments, and *n* represents the number of spacing points.

## 4. Experiment and Results

Digital instruments can compensate for the delay in piano accompaniment. Teachers use different timbres in teaching materials to express multipart music. Through listening training in the classroom, students can clearly identify timbre, sort multipart melody lines, and improve their listening skills. Adjust your learning pace to your own practice level, or use digital music aids for self-assessment. This practical training mode can form a complementary role in classroom teaching and reduce the blindness and passivity of students' extracurricular training. The experimental database consists of 1,000 music files randomly selected from the Internet music platform, including 5 music styles (pop music, folk music, light music, jazz, and classical music). The music style classification method based on the FP_Growth association rule mining algorithm is compared with the KNN algorithm and Apriori algorithm. The comparison results of the execution time of the three methods are shown in Figure 3.

It can be seen that with increasing support, the execution time of the three methods gradually decreases. However, when the support degree is small, the music style classification method proposed in this article has obvious efficiency advantages. When the minimum support degree is 0.2%, the running time of this method is about 33% of the other two methods. This is because the music style classification method based on the FP_Growth association rule mining algorithm only scans the database twice when the support is low, that is, the I/O cost is low, while the other two methods will change the option set with the length of the option set and increase the I/O overhead. The accuracy comparison results of the three music style classification methods are shown in Table 1 and Figure 4.

The classification accuracy of the music style classification method based on the FP Growth association rule mining algorithm is increased by about 2.2 percent when compared to the other two methods, as can be seen. This article does not take into account augmented chords because they are not frequently used in western music. Many academics disregard decreasing chords because they are not necessary or convenient for their research. The three main categories of major chords, minor chords, minus chords, and 36 chords, according to their names, are defined in this article for each scale. The model's output also includes a text file that contains information about each frame signal's chord type and chord boundary. The recognition rate is calculated by comparing the output chord symbol information with the actual chord symbol and dividing it by the total number of frames in the song. The newspaper chose three songs in a range of styles as the test data. The final identification results are shown in Table 2.

It is found that most errors occur in empty chords, especially in some fast-paced time periods. Because the analysis window is deterministic, if a fast-paced segment is input, it means that the window will span more notes, and a data frame is likely to contain multiple chord types, which will confuse the system. In western music, the transfer between them is very common. C major chord is also the tonic of the F minor chord, so the transition frequency from C major chord to F minor chord is also very high. Therefore, the state of the chord does not change in consecutive frames, which makes it very likely that it will transition from itself.

The diagonal vector in the covariance matrix of major chord C is also consistent with music theory.  Figure 5 shows the covariance vector of chords in C major in HMM. Pure chord tones C, E, and G have high autocorrelation, while D#, F#, and G# have low autocorrelation. Therefore, it is difficult to compare directly with other researchers' chord recognition systems. But one thing is certain: with the increase of training data, the system will get better recognition results.

Openness is the foundation of diversity, and diversity can only be achieved through openness. Solfeggio teaching should meet the needs of students' social development, scientific development, and development and strengthen students' diversified goals. To construct a multicultural learning system, while learning western classics, we should deepen our recognition of Chinese folk art, understand the cultural background and historical knowledge of popular music, and meet the requirements of curriculum standards. The rational thinking of music can start with the filling and creation, change, and repetition of phrases, which can not only cultivate students' musical sense but also cultivate students' creative thinking. Through singing solfeggio, writing dictation, improvisation, composition, memory, listening, conducting, rhythm, basic music theory, and other practices, students' comprehensive music quality has been comprehensively improved.

The pitch and overtone of the musical instrument sound source are relatively stable in the whole music area, but the singing voice is different. There are obvious pitch changes between different areas, such as vowels, consonants, and stops. There is an obvious difference. Vowels are filtered by formants for broadband excitation. However, regardless of the frequency resolution, the harmonic energy is always concentrated in the narrow bandwidth of harmonic frequency, and the distribution of edge information has not changed, but the observation mode has changed. Therefore, under the high-resolution STFT transform, the harmonic sound source is separated from the music signal. In the next experiment, several real music data were selected. Figures 6 and 7 are comparison tables of the separation performance of two real music pieces. The background music of these two songs contains rich information on harmonic sources. Among them, SDR, SIR, and SAR are Source-to-Distortion Ratio, Source-to-Interference Ratio, and Source-to-Artifacts Ratio, respectively.

It is clear that there has been a significant improvement in the separation of music and singing, particularly in the SIR performance index of singing. This demonstrates how the addition of harmonic source separation enhances the functionality of music separation by further separating the human voice from music. Due to the harmonic source separation algorithm's separation of the music and removal of some singing information, both the SIR and SAR performance indices of the background music and singing voice have decreased. Songs' harmonic information will take center stage. The harmonic source separation algorithm degrades the separation performance of music and songs because it separates a significant amount of song information from the music in the sound source. The performance of the entire music separation algorithm will be improved by improving the harmonic source separation algorithm's ability to recognise music and singing information.

Solfeggio is a fundamental and significant subject in the teaching of solfeggio. Teachers who use the piano as a teaching tool for this style of instruction will undoubtedly discover that there is only one training timbre and they must play it repeatedly, leaving them with no time to consider the issue of students' learning efficiency. At the same time, because the synthesised content is accurate in pitch and rhythm and can be played at will, bar by bar and sentence by sentence, the teachers' demanding work of continuous accompaniment and fan singing can be lessened in the context of solfeggio training. The presentation sound can be changed at random, depending on the audience, teachers, and students. A single melody can be gradually layered in complex orchestral works, or the appearance of all parts can be gradually reduced. This allows for thorough teaching of music analysis to students. The speed and accuracy with which the computer completes these tasks enhance and save classroom time, increase classroom utilisation, and enhance the effectiveness of instruction.

## 5. Conclusions

The use of digital musical instruments, sound systems, and other technologies in the teaching of music theory has been encouraged by the application and advancement of DM technology, which has also expanded classroom teaching avenues and improved classroom lesson materials. The uneven distribution of educational resources, inability to adapt intelligently, and other issues are successfully resolved by the music curriculum model based on DM technology, which effectively utilises the music education information platform architecture of the education cloud and DM technology. In music style classification methods, the FP Growth association rule DM method is more prevalent and outperforms all others. The situation of sound sources in music is analyzed using sound source type analysis technology, and the residual information is separated accordingly. According to experimental tests, residual disturbing sound sources in singing information are significantly diminished, and the overall quality of separated music is also improved.

## Figures and Tables

**Figure 1:** DM interactive information management system architecture.

**Figure 2:** Frame diagram of the string recognition system.

**Figure 3:** Running time comparison.

**Figure 4:** Classification accuracy comparison curve.

**Figure 5:** Large C chord covariance vector.

**Figure 6:** Song 1 separation performance comparison.

**Figure 7:** Song 2 separation performance comparison.

**Table 1:** Classification accuracy.

Music style type	Methods of this article	KNN	Apriori
Pop music	85.63	81.21	83.25
National music	68.71	60.33	62.04
Light music	69.08	65.58	66.98
Jazz	80.11	77.12	74.52
Classical music	69.32	63.09	64.33

**Table 2:** Chord recognition result.

Music style type	Length	Recognition (%)	Average recognition rate (%)
Pop music	8.06 seconds/41 frames	82.33	78.2
National music	20 seconds/669 frames	78.21	
Light music	15 seconds/641 frames	74.06	

## Data Availability

The data used to support the findings of this study are available from the corresponding author upon request.
